This article has been retracted.

# Nursing Research on Benign Prostatic Hyperplasia Based on Continuous Nursing Care

**DOI:** 10.1155/2022/9855770

**Published:** 2022-07-04

**Authors:** Shasha Li, Ying Sun, Jie Liu, Fei Han, Bingwen Liu, Wanqing Liu

**Affiliations:** ^1^Department of Geriatrics, The Sixth Hospital of Wuhan, Affiliated Hospital of Jianghan University, China; ^2^Department of Urology, Wuhan No.1 Hospital, China; ^3^Department of Nephrology, People's Hospital of Dongxihu District, China

## Abstract

**Purpose:**

To explore the nursing research of prostatic hyperplasia based on continuous nursing and based on the combination of medical care and nursing.

**Methods:**

A prospective study of 96 patients with benign prostatic hyperplasia admitted to our hospital from November 2019 to May 2021 was selected. According to the random number table method, they were divided into an observation group and a control group with 48 cases each. The control group used routine nursing and discharge guidance, and the observation group implemented continuous care based on the combination of medical care and nursing on the basis of the control group. The differences in the scores of quality of life, self-care ability, quality of life score, and sleep quality were compared between the two groups.

**Results:**

After 3 months of nursing, the quality of life scores (health status, psychology, social relationship, environment, physiology, and quality of life scores) of the observation group was higher than those of the control group (*P* < 0.05). After 3 months of nursing, the quality of life scores of disease, physiology, society, psychology, and satisfaction of the observation group was significantly higher than those of the control group, which was statistically significant (*P* < 0.05). After 3 months of nursing, the observation group's sleep quality scores in all dimensions (time to fall asleep, sleep time, sleep quality, sleep efficiency, hypnotics, sleep disorders, and day disorders) were higher than those of the control group (*P* < 0.05). After 3 months of nursing, the observation group's self-care skill score, self-responsibility score, health knowledge score, and self-concept score were better than those of the control group (*P* < 0.05).

**Conclusion:**

Continued nursing care based on the combination of medical and health care for prostate hyperplasia is beneficial to improve sleep quality and improve the patient's quality of life score and self-care ability and provide certain references for clinical care of patients with benign prostatic hyperplasia.

## 1. Introduction

Prostatic hyperplasia is the most common benign disease that causes urinary dysfunction in elderly men. It increases with age, and the incidence rate is greater than 50% by the age of 60 [1]. The main clinical manifestations are overactive bladder, obstructive symptoms, and related complications [2]. These symptoms have varying degrees of impact on the patients' sleep, activities of daily living, social activities, etc., leading to depression, anxiety, and other psychology of the patients [3]. Because benign prostatic hyperplasia is a progressive disease, many patients still need surgical treatment to solve lower urinary tract symptoms. Studies have proved that surgical treatment is one of the effective methods to treat benign prostatic hyperplasia, which is beneficial to improve the quality of life of patients [4]. Due to the long course of benign prostatic hyperplasia, which seriously affects the quality of life and sleep quality of patients, increases the mental pressure of patients, and causes their physical and mental pain, how to formulate scientific nursing measures to improve the quality of life of elderly patients with benign prostatic hyperplasia is a top priority [5]. The integration of medical care and care emphasizes the integration of existing resources under the overall planning of the government, and professionally trained medical staff provides medical treatment, rehabilitation, life care, psychological counseling, and hospice care for elderly patients with chronic diseases and semidisabled, disabled, and advanced tumors. The integrated service model, etc., has been promoted and applied in the care of a variety of chronic diseases [6]. Continuing care under the integrated medical care model can extend the hospital's care of patients to the community, family, or after they are discharged, so that the hospital beds can be better recycled [7]. Rehabilitation care technology of life care personnel in China has been improved, and the long-term health service needs of elderly patients with chronic diseases have been met. However, the application and empirical analysis of continued care in elderly patients with benign prostatic hyperplasia under the integrated medical care model have not been reported yet [7]. Based on this, this study explores the nursing research of prostatic hyperplasia based on the continuation of medical care. The current research report is as follows.

## 2. Materials and Methods

### 2.1. Research Object

We selected 96 patients with benign prostatic hyperplasia admitted to our hospital from November 2019 to May 2021 as a prospective study. The screening process is shown in Figure 1.According to the random number table method, they were divided into an observation group and a control group, each with 48 cases. The patients were 62-85 years old, both volunteer to participate in this study and sign the relevant consent form. According to the Prostate Symptom Score (IPSS), patients were scored from 4 to 19 points. The clinical symptoms were various degrees of frequent urination, urgency, and dysuria. Patients with malignant tumors and other urinary system diseases were excluded. There were 48 patients in the observation group, with the ages of 63-86 years old, with an average age of 68.13 ± 9.85 years old, and the course of disease was 1 to 17 years, with an average course of 12.54 ± 2.86 years; patients in the control group were aged 61-82 years with an average age of 61.64±6.37 years old, and the patient's course of illness was 2-17 years, with an average course of 10.25 ± 2.33 years. The observation group and the control group had no statistically significant differences in general clinical data, such as age, course of disease, and education level, (*P* > 0.05), and they had good comparability (*P* > 0.05).

### 2.2. Inclusion and Exclusion Criteria

Inclusion criteria were as follows: (1) The included patients meet the “Prostate artery embolisation for benign prostatic hyperplasia: a systematic review and meta-analysis” diagnostic criteria for benign prostatic hyperplasia, have clear consciousness and elementary school education and above, with no mental and language disorders, able to compare, a good communicator, and perform transurethral resection of the prostate in our hospital [8]; (2) for patients diagnosed with benign prostatic hyperplasia in our hospital, the patient can actively cooperate with the treatment and nursing work, and the compliance is good. The patient agrees to this study and signed the informed consent; and (3) patients who have undergone transurethral prostatic hyperplasia resection and generally have complete information and clear consciousness, have reading and language skills, and voluntarily participate in this study. Exclusion criteria were as follows: (1) We excluded patients with mental disorders, with physical disorders, such as heart and kidney functions, and who are not physically fit to participate in this study; (2) patients with life expectancy ≤6 months and deafness due to aphasia and who cannot communicate and meet the diagnostic criteria for Alzheimer's; and (3) patients with poor general conditions of urinary tract tumors, with mental disorders who cannot cooperate, and who cannot obtain follow-up results.

### 2.3. Intervention Methods

The control group adopts routine nursing and discharge guidance, that is, ① the patients should be evaluated for nursing, that is to say, the appropriate nursing plan should be formulated for the patient according to the patient's condition and various aspects of the physical condition. Secondly, give the patients some basic nursing interventions, especially pay attention to the morning and evening care and clean care of the patients. On the one hand, it can maintain the hygiene of the patients and can effectively avoid secondary infections caused by bacteria. ② Because the treatment process of patients with benign prostatic hyperplasia is relatively long, it is inevitable that some negative emotions such as anxiety will appear during the treatment. Therefore, nursing staff should strengthen the communication with patients, eliminate patients' negative emotions in time, and tell patients that disease was successfully cured by the pathology of the hospital to increase patients' confidence in treatment. ③ Among the patients admitted to the hospital, most of them do not know enough about the disease of prostate hyperplasia. Therefore, nursing staff should carry out health education to patients, including the causes and mechanisms of prostate hyperplasia and precautions, so that patients can fully understand their symptoms, so as to ensure that patients can reduce their anxiety during the treatment process. One-step treatment provides convenience. ④ Prostatic hyperplasia has a relatively large impact on the life of patients and often leads to a decline in the quality of life of the patients, especially in terms of the patient's work and rest time and sleep quality.

On the basis of the control group, the observation group carried out continuous care based on the combination of medical care and nursing, that is, ① 2 hours before the operation, the advantages of surgical treatment, the operation method, and the operation process were explained to the patient, and oxygen inhalation 2~4 L/min will be given if necessary; no eating or drinking is allowed within 6 hours postoperative, and then you can enter a liquid diet and turn over and knock the back every 3 to 4 hours. After removing the pillow and lying supine for 6-8 hours, the head was turned to one side to prevent malignant vomiting caused by anesthesia and to keep the airway unobstructed. ② Before discharge, the nurse in charge instructs the patient to do anal contraction exercises, instructs them to exercise 3 times, in the morning, noon, and evening, and do 100 consecutive contraction exercises each time, not less than 30 s each time, and instruct patients to avoid sex, lifting heavy objects, and long-distance walking within 6 weeks, avoid more intense exercise within 3 months, and maintain a comfortable mood, strengthen self-management, observe and record the number of urination, urine color, and urine line daily, and review regularly. According to the actual situation of the patient, guide diet, quit smoking and alcohol, drink 2000 mL daily to increase urine output and prevent urine concentration. ③ After discharge, the patient is advise to carry out community care in the community, under the guidance of urology specialists and nurses in charge, community nurses and nurses in attendance. Nurses in charge instruct patients to do anal contraction training 10 times a day, perform bladder function training, drink water according to the plan, repeatedly contract the anus, relieve smooth muscle contraction, gradually extend the time of urination, adjust prostate function, and make records; organize health education meetings and health lectures every Thursday at 14 : 00; and invite patients and their families to participate, share their experiences, and adopt positive psychological counseling to improve the mood of patients and promote their recovery. On the basis of routine care, nurse in charge carry out the continuous nursing plan under the combined medical care and nursing care every day and make a record, including 3 warm reminders for taking medications, 1 radio gymnastics activity, 25 minutes each time, psychological assessment and considerate comfort care for the patient 1 time a day, and serve with a smile. Daily room cleaning is performed once a day, perineum and urinary tract cleaning are performed in the morning and afternoon each day, and blood pressure and body temperature are measured once each.

### 2.4. Observation Indicators

#### 2.4.1. Quality of Life Score

The patient will be followed up by telephone after 3 months of care, and the quality of life score will be performed.

In this study, the World Health Organization Quality of Life Assessment Scale was used to evaluate the quality of life of elderly patients with benign prostatic hyperplasia. The main content includes 6 dimensions of quality of life, physiology, psychology, health, environment, and social relations, with a total of 26 items. Each item uses the Likert five-level scoring method, from “very poor” to “very good,” respectively, 1 to 5 points. The higher the score, the better the patient's postoperative quality of life. The Cronbach coefficient of this scale is 0.754.

#### 2.4.2. Quality of Life

*(1) Beta Version of the Quality of Life Scale for Patients with Benign Prostatic Hyperplasia (BPHQLS)*. This scale is suitable for measuring the quality of life of patients with benign prostatic hyperplasia in my country during the first two weeks when they are tested. This table has 74 items in total. There are 5 dimensions: disease (27 items), physiology (16 items), society (13 items), psychology (10 items), satisfaction (8 items). In this study, the Cronbach's coefficient of the scale was 0.96.

#### 2.4.3. Sleep Quality

After 3 months of patient care, the Pittsburgh Sleep Quality Questionnaire was used to evaluate the postoperative sleep quality of patients with benign prostatic hyperplasia. There are 7 dimensions and 18 items in total. Each item adopts the Likert 4-level scoring method, from “very good” to “very poor,” respectively, 0 to 3 points. The higher the score, the worse the patient's postoperative sleep quality. Cronbach's coefficient of this scale is 0.817.

#### 2.4.4. Self-Care Ability

Compare the self-care ability scores of the two groups of patients using the self-care ability measurement scale to evaluate before the intervention and 3 months after the intervention, including 4 items of self-care skills, health knowledge, and self-concept and self-responsibility. There are a total of 43 items, each item scores 0-4 points, and the total score is 172 points. The higher the score, the stronger the patient's self-care ability.

### 2.5. Statistical Methods

Use Epidata to enter all the data, and then use SPSS 25.0 to statistically process the data. The data needs to be entered into the computer database by a second person to ensure the completeness and accuracy of the data. The measurement data was expressed as mean ± standard deviation ($\bar{x}\pm S$) using *t*-test, statistically *P* < 0.05 is meaningful.

## 3. Results

### 3.1. Comparison of Quality of Life Scores

After 3 months of nursing, the quality of life scores (health status, psychology, social relationship, environment, physiology, and quality of life scores) of the observation group was higher than those of the control group (*P* < 0.05), see Table 1.

### 3.2. Comparison of Quality of Life Scores

After 3 months of nursing, the quality of life scores of disease, physiology, society, psychology, and satisfaction of the observation group was significantly higher than those of the control group, which was statistically significant (*P* < 0.05), see Table 2.

### 3.3. Comparison of Scores in various Dimensions of Sleep Quality

After 3 months of nursing, the observation group's sleep quality scores in all dimensions (time to fall asleep, sleep time, sleep quality, sleep efficiency, hypnotics, sleep disorders, and day disorders) were all higher than those of the control group, which were statistically significant (*P* < 0.05), see Table 3.

### 3.4. Comparison of Self-Care Ability Scores

After 3 months of nursing, the observation group's self-care skill score, self-responsibility score, health knowledge score, and self-concept score were better than those of the control group (*P* < 0.05), and the comparison was statistically significant (*P* < 0.05) (Table 4).

## 4. Discussion

Continuing care is especial for patients who have a higher readmission rate or still have a higher need for care after discharge [9]. Foreign surveys show that discharge patients have the most urgent need for continuity care before and within 2 weeks after discharge. Continued care under the concept of the integration of medical care and nursing can greatly improve the satisfaction of elderly patients with chronic diseases in nursing service and the rate of compliance with doctor's orders, reduce the rate of secondary admissions, and improve the quality of life [10]. Through continued care, it can provide long-term, effective, and remote guidance and management for elderly care for the elderly, enhance the professionalism and pertinence of nursing services, and improve the quality of life and physical and mental health of the elderly [11].

After 3 months of nursing in this study, the quality of life scores (health status, psychology, social relationship, environment, physiology, and quality of life scores) of the observation group was higher than those of the control group, indicating that continued nursing under the medical-care integration mode was significantly improved together with the overall quality of life in elderly patients with benign prostatic hyperplasia after surgery. Specific reasons were as follows: It may be related to the implementation of disease-specific and individualized treatment and care for elderly patients with benign prostatic hyperplasia. It is recommended that professional medical institutions and elderly care institutions develop closer counterpart cooperation, strengthen the integration of medical, rehabilitation, elderly care, and nursing resources, promote active participation of elderly patients in social activities, and further improve the quality of life of elderly patients with prostate hyperplasia in elderly care institutions [12].

After 3 months of nursing in this study, the scores of all dimensions of sleep quality (time to fall asleep, sleep time, sleep quality, sleep efficiency, hypnotics, sleep disorders, and day disorders) of the observation group were higher than those of the control group. It shows that continued nursing under the mode of integrated medical care can significantly improve the sleep quality of elderly patients with benign prostatic hyperplasia. On the one hand, continuous care under the combined medical care model not only pays attention to the physiological aspects of elderly patients with benign prostate hyperplasia but also improves the health and rehabilitation of elderly patients with benign prostate hyperplasia from a psychological and social perspective, thereby improving the patient's sleep quality [13]. On the other hand, professional nursing measures help the recovery of elderly patients with benign prostatic hyperplasia and improve their physiological functions. In addition, community nurses use their professional knowledge to guide the healthy diet and reasonable exercise of elderly patients with benign prostatic hyperplasia and choose appropriate personal lifestyles for them, so that they can live healthy and happily everyday [14]. This is not only the expectation of the vast majority of elderly patients but also a prerequisite for good health. It is recommended that in future research and implementation plans, more attention should be paid to the use of scientific methods to improve the sleep quality of elderly patients with prostate hyperplasia in elderly care institutions [15].

After 3 months of nursing in this study, the observation group's self-care skill score, self-responsibility score, health knowledge score, and self-concept score were better than those of the control group. The reason for the analysis may be that the initial period of most patients returning to the family after discharge is a dangerous period when treatment cannot be continued well or some potential adverse events are prone to occur. Therefore, self-care ability is low. Early follow-up of patients with benign prostatic hyperplasia and the development of corresponding evaluation forms and care plans optimize the health of patients after transfer from the hospital to home [16–19]. Self-care theory believes that the purpose of nursing is to guide patients how to self-care in their daily lives by providing specific and detailed nursing guidance to patients, reducing the use of health resources, and at the same time promoting the healing of diseases [20]. Hospital medical staff and related care providers should not regard patient discharge as the end of their responsibilities for treatment and care of patients but should try to provide patients with safe and effective transition care [21].

After 3 months of nursing in this study, the quality of life scores of disease, physiology, society, psychology, and satisfaction of the observation group was significantly higher than those of the control group, which was statistically significant. It shows that continual nursing can improve the quality of life of elderly patients with benign prostatic hyperplasia. The evaluation of quality of life can better understand the patient's feelings about the disease. It plays an important role in the improvement of treatment and nursing methods and in evaluating the effectiveness of curative effects. This study is similar to the results of several studies on continuity nursing in Hong Kong, my country. The connotation of quality of life not only refers to the body's physical absence of disease but also includes psychological balance and social interaction in a sound state [22]. As the age increases, the symptoms of patients become more obvious. If they do not receive good care after returning home from the hospital, or do not understand self-care, the quality of life will be affected [23–25]. Continuing care takes personalized nursing measures to cultivate their independent ability by strengthening the maintenance of the relationship between medical staff and patients and the integration of medical services [24]. Learn self-care and self-care in daily life, enhance their self-confidence to maximize their physical and mental state, reduce dependence on family members and excessive use of medical resources, and the quality of life will also improve [26–28].

The construction of a continuous nursing model based on the concept of the integration of medical care and elderly care, combined with medical care and elderly care services, helps to improve the treatment compliance of the elderly, improve the clinical and physiological indicators, reduce the number of rehospitalizations, and improve the happiness and social welfare of the elderly [29, 30], supporting the quality of life, while improving service quality [31, 32]. At present, “hospital-” continuation care is still in its infancy, and there are many factors that affect the smooth implementation of continuation care. Therefore, under the premise of perfecting the reform of my country's medical system, drawing on the experience of foreign continuation of nursing, further strengthening the professional quality of nursing staff, establishing a multidisciplinary and multiprofessional team continuance nursing model service, embodying continuity of humanistic nursing, and striving to explore suitable for China, the continuity of care model achieves a healthy and aging population [33, 34].

This study provides reliable experience in the care of discharged patients after radical prostatic hyperplasia in our hospital. It also promotes the improvement of the quality of care in our department to a certain extent, while still having certain limitations: first of all, this study is inevitable due to the limitation of the number of cases. There will be some shortcomings. Secondly, the sample size of this study is small. Due to the influence of different factors, such as age and education level, most of the patients are rural elderly patients, who have poor grasp of disease knowledge and low cognition. Therefore, the intervention group has relatively few samples. Finally, the intervention time is short, and the continuity of nursing measures needs to be further improved in the future. In the future, it is necessary to strengthen the promotion of network platforms, expand the sample size, and extend the intervention time. To sum up, the continued care of BPH based on the combination of medical care and nursing is beneficial to improve the quality of sleep and improve the patient's quality of life score and self-care ability and provide a certain reference for the clinical care of BPH patients.

## Figures and Tables

**Figure 1:** Patient screening flowchart.

**Table 1:** Comparison of quality of life scores between the two groups ($\bar{x}\pm s$).

Group	Health status	Psychology	Social relationship	Environment	Physiological	Quality of life
Observation group (48)	13.64 ± 2.31	10.49 ± 3.24	14.27 ± 2.14	11.27 ± 2.23	3.21 ± 0.31	3.54 ± 1.16
Control group (48)	7.68 ± 1.47	6.89 ± 1.66	4.23 ± 0.57	7.25 ± 1.82	2.23 ± 0.57	1.83 ± 0.45
*t*	15.081	6.851	31.409	9.676	10.464	9.522
*P*	0.000	0.000	0.000	0.000	0.000	0.000

**Table 2:** Comparison of quality of life scores between the two groups ($\bar{x}\pm s$).

Group	Disease	Physiological	Society	Psychology	Satisfaction
Observation group (48)	52.16 ± 9.20	51.31 ± 8.16	52.21 ± 10.32	52.14 ± 10.29	51.27 ± 12.21
Control group (48)	45.29 ± 11.61	46.20 ± 10.52	47.23 ± 9.68	47.15 ± 12.46	46.26 ± 10.37
*t*	3.213	2.659	2.438	2.139	2.167
*P*	0.002	0.009	0.017	0.035	0.033

**Table 3:** Comparison of the scores of sleep quality in each dimension of the two groups of patients ($\bar{x}\pm s$, min).

Group	Time to fall asleep	Sleeping time	Sleep quality	Sleep efficiency	Hypnotics	Sleep disorder	Day barrier
Control group (48)	1.19 ± 0.15	1.26 ± 0.38	0.64 ± 0.17	1.86 ± 0.48	1.37 ± 0.23	1.17 ± 0.21	1.18 ± 0.32
Observation group (48)	1.92 ± 0.49	1.61 ± 0.27	1.68 ± 0.47	2.58 ± 0.61	2.65 ± 0.42	2.52 ± 0.33	1.61 ± 0.42
*t*	-9.80	-5.202	-24.030	-6.427	-18.519	-23.912	-18.763
*P*	0.000	0.000	0.000	0.000	0.000	0.000	0.000

**Table 4:** Comparison of the self-care ability scores of the two groups of patients ($\bar{x}\pm \text{s}$).

Group	Self-care skills	Self-responsibility	Health knowledge	Self-concept
Observation group (*n* = 48)	46.79 ± 6.82	29.29 ± 6.06	27.17 ± 8.43	28.94 ± 7.02
Control group (n = 48)	38.12 ± 8.43	21.87 ± 5.12	21.16 ± 7.42	23.21 ± 6.96
*t*	5.540	6.480	3.708	4.016
*P*	<0.001	<0.001	<0.001	<0.001

## Data Availability

No data were used to support this study.
